The article "An Approach to Uropathogenic Escherichia Coli in Urinary Tract Infections" was retracted in 2011. Reason: plagiarized text.

# An Approach to Uropathogenic *Escherichia Coli* in Urinary Tract Infections

**DOI:** 10.4103/0974-2727.72152

**Published:** 2010

**Authors:** K Prabhat Ranjan, Neelima Ranjan, Arindam Chakraborty, D R Arora

**Affiliations:** Department of Microbiology, Pt. B D Sharma Postgraduate Institute of Medical Sciences, Rohtak, Haryana, India; 1 Department of Microbiology, Kasturba Medical College, Mangalore, Karnataka, India; 2 Department of Microbiology, Maharaja Agrasen Medical College, Agroha, Hisar, Haryana, India

**Keywords:** *Escherichia Coli*, hemolysin, hemagglutionation, serum resistance, surface hydrophobicity, virulence factor

## Abstract

**Purpose:**

To study the occurrence and characterization of Uropathogenic *Escherichia Coli* (UPEC) in cases with urinary tract infections.

**Materials and Methods:**

A total of 220 symptomatic cases from urinary tract infections and 50 stool samples from apparently healthy individuals were included. The colonies identified as *Escherichia Coli* were screened for virulence factors, that is, hemolysin, Mannose Resistant and Mannose Sensitive Hemagglutination (MRHA, MSHA), Cell surface hydrophobicity, and Serum resistance.

**Results:**

Among the 220 cases 91 (41.36%) were hemolytic, 68 (30.90%) showed MRHA, 58 (26.36%) were cell surface hydrophobicity positive, and 72 (32.72%) were serum-resistant. In 50 controls, three (6%) were hemolytic, six (12%) showed MRHA, nine (18%) showed cell surface hydrophobicity, and 12 (24%) were serum-resistant. The difference between cases and controls for hemolysis and MRHA were significant (*P*<0.001 and *P*<0.01, respectively). A total of 14 atypical *E. coli* were isolated from the urine and all showed the presence of one or the other virulence markers. Out of the 18 mucoid *E.coli* isolated, 10 were serum-resistant.

**Conclusions:**

The present study revealed that out of 220 urinary isolates, 151 could be labeled as UPEC.

## INTRODUCTION

Urinary tract infection (UTI) is one of the most important causes of morbidity and mortality. *E.coli* is the most frequent urinary pathogen isolated from 50 – 90% of all uncomplicated urinary tract infections.[1] *E.coli* present in the gastrointestinal tract as commensals provide the pool for initiation of UTI. It has been traditionally described that certain serotypes of *E.coli* are consistently associated with uropathogenicity and are designated as Uropathogenic *E.coli* (UPEC). These isolates express chromosomally encoded virulence markers. These markers of UPEC are expressed with different frequencies in different disease states, ranging from asymptomatic bacteriuria to chronic pyelonephritis.

In the late 1970s, it was recognized for the first time that *E.coli* strains causing urinary tract infections typically agglutinate human erythrocytes, despite the presence of Mannose,[2] and this was mediated mainly by fimbriae. Subsequently an array of virulence factors were proposed as virulence markers for uropathogenic isolates of *E.coli*. It is now recognized that there are a subset of fecal *E.coli* having the above-mentioned factors that can colonize the periurethral area, enter the urinary tract, and cause symptomatic disease. These are currently defined as UPEC.[3]

However, most of these studies have been carried out on patient isolates and no studies have been carried out on commensal / gut isolates. In addition, the relative importance of these bacterial factors has not been validated. In the present study an attempt has been made to answer these two questions with respect to four proposed virulence factors namely hemolysin, hemagglutination, cell surface hydrophobicity, and serum resistance.

The article "An Approach to Uropathogenic Escherichia Coli in Urinary Tract Infections" was retracted in 2011. Reason: plagiarized text.

## MATERIALS AND METHODS

### Samples

The study was conducted in the Department of Microbiology, Maharaja Agrasen Medical College. Urine samples from a total of 220 *E. coli* from all age groups of symptomatic cases of UTI, belonging to the Departments of Urology, Nephrology, Medicine, and Pediatrics were studied for the detection of virulence markers. A total of 50 fecal isolates from apparently healthy individuals who had come for a routine health checkup were screened for *E. coli* and studied further for virulence markers and included as controls. Urine samples were processed as per standard protocol.[4] Lactose fermenting colonies on MacConkey’s agar (MA) showing significant bacteriuria (10^5^ CFU/ml) were processed and identified as *E. coli* by standard biochemical tests.[5] Standard uropathogenic *E. coli* serotypes O4 and O6 and *E.coli* ATCC 25922 were used as controls for detection of the virulence markers. The additional features noticed in terms of colony morphology were, whether they were mucoid / non-mucoid and the biochemical reactions, whether they showed hemolysis on sheep blood agar after incubation overnight, and whether they were typical or atypical isolates. An isolate was considered as typical if it was a lactose fermenter and aerogenic and atypical if it was a non-lactose fermenter and anaerogenic. *E. coli* thus obtained from cases with significant counts (10^5^ CFU/ml) were screened for virulence markers.

### Detection of virulence factors

#### Hemolysin production

The plate hemolysis test was done for the detection of α-hemolysis produced by the *E. coli*.[6] The bacteria were inoculated into 5% sheep blood agar and incubated overnight at 35°C. Hemolysin production was detected by the presence of a zone of complete lysis of the erythrocytes around the colony and clearing of the medium.

The article "An Approach to Uropathogenic Escherichia Coli in Urinary Tract Infections" was retracted in 2011. Reason: plagiarized text.

#### Hemagglutination

*E. coli* grown on Mac Conkey agar plates were inoculated into 5 ml of phosphate buffered saline pH 7.4 (PBS) and incubated for five days at 37°C, to obtain fimbriae *E. coli*. The pellicle that formed on the surface was noted and subcultured onto a colonization factor antigen (CFA) agar; 0.5 ml of fresh group A-positive blood was obtained from the blood bank and added to an equal amount of Alsever’s solution. This was washed thrice and 3% erythrocyte suspension was prepared with PBS. The colonies of *E. coli* growth on CFA were emulsified on a VDRL slide in PBS, to form a milky white suspension. To this an equal volume of 3% suspension of erythrocytes was added and gently mixed with a wooden applicator. The slide was rotated manually for three to five minutes, observed for hemagglutination macroscopically, within 10 minutes. To determine the mannose-resistant hemagglutination, colonies from the CFA were emulsified on a slide in PBS. A drop of 2.5% of mannose was added. To this mixture, an equal volume of 3% suspension of erythrocytes was added and gently mixed with a wooden applicator. The slide was rotated for three to five minutes and observed for hemagglutination (HA). Hemagglutination was designated as a mannose-resistant hemagglutination (MRHA) if the HA was observed with and without mannose to the same degree, and mannose sensitive hemagglutination (MSHA) if HA was inhibited in the presence of mannose.[6] The following controls were used: *E. coli* ATCC 25922 for MSHA. UPEC serotypes 06 and 011 for MRHA.[5]

#### Cell surface hydrophobicity

The cell surface hydrophobicity of *E. coli* was determined by the salt aggregation test (SAT).[6,7] One loopful (10 µL) of bacterial suspension made in phosphate buffer was mixed with an equal volume of ammonium sulfate solution of different molarity, that is, from 0.3125 m through 5.0 m, on a glass slide and observed for one minute, while rotating. The highest dilution of ammonium sulfate solution, giving a visible clumping of bacteria, was scored as the salt aggregation test (SAT) value. Strains showing aggregation in 0.002 m phosphate buffer alone (pH 6.8) were considered to be auto aggregative. *E. coli* strains that had a SAT value ≤ 1.25 m were considered hydrophobic.[6,7]

#### Serum resistance

Serum resistance was studied using a fresh culture of the isolates.[6,7] Overnight cultures of *E. coli*, grown at 37°C on blood agar, were harvested and the cells were suspended in Hank’s balanced salt solution (HBSS). The bacterial suspension (0.05 mL) was incubated with serum (0.05 mL) at 37°C for 180 minutes. Ten microliters of samples were withdrawn and spread on blood agar plates, which were then incubated at 37°C for 18 hours and the viable count was determined. Resistance of bacteria to serum bactericidal activity was expressed as the percentage of bacteria surviving after 180 minutes of incubation with serum, in relation to the original count. Bacteria were termed serum sensitive, if the viable count dropped to 1% of the initial value, and resistant if >90% of the organisms survived after 180 minutes.

The article "An Approach to Uropathogenic Escherichia Coli in Urinary Tract Infections" was retracted in 2011. Reason: plagiarized text.

### Statistical Analysis

The chi square test was used to compare the occurrence of virulence markers in both the cases and controls. P value less than 0.05 was considered significant.

## RESULTS

A total of 220 *E. coli* were isolated from the urine samples, from UTI. Out of these, 191 samples had significant bacteriuria with counts 10^5^ CFU/mL and 29 had probably significant bacteriuria with counts between 10^4^ and 10^5^ CFU/mL.

### Phenotypic and biochemical characteristics of *E. coli*

A total of 18 *E. coli* isolates were mucoid lactose fermenting colonies. All controls were non-mucoid lactose fermenters. Out of 220 isolates 14 were non-lactose fermenters and anaerogenic and considered as atypical *E. coli*.

### Virulence markers of Uropathogenic *E. coli* obtained from cases and controls

The performance of the standard uropathogenic *E. coli* (UPEC) isolates was satisfactory in all the four assays. Occurrence of UPEC with virulence markers in different combinations among cases and controls.

### Hemolysin

Among the 220 cases 91 (41.36%) were hemolytic. Among 50 controls, three (6%) were hemolytic. The difference between the cases and controls, for hemolysin production, was highly significant (*P*<0.001).

### Hemagglutination

A total of 68 (30.90%) among 220 cases and six (12%) among 50 controls showed mannose-resistant hemagglutination. There was a significant (*P*<0.01) difference in MRHA between cases and controls.

### Cell surface hydrophobicity

A total of 58 (26.36%) among 220 cases and nine (18%) among 50 controls were cell-surface hydrophobic. There was no significant difference (*P*>0.05) between the cases and controls, for cell surface hydrophobicity.

### Serum resistance

Among 220 cases, 72 (32.72%) *E. coli* were serum-resistant and among 50 controls, 12 (24%) *E. coli* were serum-resistant. There was no significant difference (*P*>0.05) in the cases and controls for serum resistance. The results of virulence markers among *E. coli* isolates from cases and controls.

### Atypical / Mucoid *E. coli* and virulence

Of the 18 mucoid lactose fermenters, 10 were serum-resistant and three were hemolytic, two were MRHA, and one was MSHA. Among the 14 non-lactose fermenters, all had one or more virulence markers.

The article "An Approach to Uropathogenic Escherichia Coli in Urinary Tract Infections" was retracted in 2011. Reason: plagiarized text.

## DISCUSSION

Considering the high degree of morbidity and mortality of UTIs, the subject of uropathogenic *E. coli* was receiving increasing attention. Cell morphology and molecular biology studies have revealed that uropathogenic *E.coli* express several surface structures and secrete protein molecules, some of them cytotoxic and peculiar to the strains of *E. coli*, causing UTI.[1] Hence, it is important to identify UPEC from non-UPEC isolates in the urinary samples. Results in this study showed that most of the urinary isolates from cases had more than one virulence marker. In this case-control study we conclude that UPEC strains are definitely associated with the aetio-pathogenesis of UTI. The occurrence of multiple virulence factors in the UPEC strains further strengthens the concept of the association of UPEC with urinary pathogenicity. It was interesting to note that UPEC with multiple virulence factors were significantly more in the cases than in the controls.

Phenotypic and biochemical characterization revealed interesting findings. A total of 18 urinary isolates were mucoid and all these were obtained from the cases only. No mucoid strains were isolated from the control group. Furthermore, 10 of these 18 were serum-resistant. The mucoid strains were capsulated[8] and the capsule conferred serum and phagocyte resistance to some *E. coli* strains.[3] This property was attributed to the content of sialic acid, which reduced the ability of the bacterial surface to activate and complement by an alternative pathway. However, eight mucoid strains were susceptible to the serum indicating that non-capsular factors had a role in serum resistance. Thus, the conventional phenotypic marker, such as the capsule, was also an important virulence factor for the UPEC. In the present study, 14 (6.36%) of the 220 isolates were atypical *E. coli*. Altered phenotypes could be due to an altered genetic makeup. Bhat *et al*.[9] studied 210 *E. coli* strains isolated from the urine and found 26 (12.4%) to be atypical. In their study of the 26 atypical urinary isolates, 12% were hemolytic and three had hydrophobicity (< 0.156) and were MRHA positive and all the atypical *E.coli* had one or the other virulence marker, indicating that an atypical phenotype probably contributed to their virulence. The cytolytic protein toxin secreted by most hemolytic *E.coli* strains was α-hemolysin. *E.coli* also produced cell-associated lysin on blood agar plates and hemolysin caused a clear zone of lysis.[10] In the present study, although the nature of hemolysin was not further characterized it could be considered as a cytotoxic necrotizing factor (hemolysin). The difference between cases and controls for the production of hemolysin was highly significant (*P*<0.001). This was similar to the Johnson *et al*.[2] study, where hemolysin was produced by 38% of the urinary isolates and 12% of the fecal isolates. Hemagglutination was mediated by the fimbriae.[11] MRHA could be mediated by P fimbriae. Thus, the MRHA positive strains could be considered as UPEC, most likely having P fimbriae.[2] In the present study there was a significant difference in MRHA between cases and controls (*P*<0.01). This was similar to a study by Johnson[2] *et al*, where 58% of the urinary isolates and 19% of the fecal isolates showed MRHA. The expression of type 1 fimbriae was indicated by MSHA. MSHA were more in the fecal strains than in urinary isolates, in our study. More work is required to assess the role of MSHA in pathogenecity. The role of the cell-surface hydrophobicity in mediating bacterial adherence to mammalian cells was conceived by Mudd and Mudd.[12] Crystalline surface layers: the ‘S’ layer present on both gram negative and gram positive organisms play a role in this.[13] Hydrophobicity is a recently described novel virulence mechanism by *E. coli*. In the present study, although there was no significant difference in cell-surface hydrophobicity between the cases and controls (*P*>0.05), more isolates from the cases were hydrophobic. Taylor[14] reviewed that bacteria were killed by normal human serum through the lytic activity of an alternative complement system. Bacterial resistance to killing by serum, results from the individual or combined effects of the capsular polysaccharide, O polysaccharide, and surface proteins.[15] Although more *E. coli* isolates from the cases were serum-resistant compared to the controls, the difference was not statistically significant (*P*>0.05). The O group designation reveals little about a strain. The apparent virulence associated with certain groups may be mediated through other virulence factors like P fimbriae, hemolysin, and serum resistance, which is commonly associated with UTI-associated strains.[2]

In this study, 151 out of 220 isolates had one or more virulence factors. When a comparison was done between the urinary and fecal *E.coli* isolates, hemolysin production, presence of capsule, and the capacity to cause MRHA, emerged as important virulence factors. The hemolysin, especially α-hemolysin, also known as cytotoxic necrotizing factor, is strongly proinflammatory leading to secretion of IL-6 and chemotaxins, which sets pace for the pathogenesis of renal disease. The capacity to cause MRHA is due to various adhesions mainly P fimbriae, P-associated fimbriae, and FIC fimbriae, seen in pyelonephritis cases. These adhere to the fibronectin on the uroepithelial cells contributing to the persistence.

The article "An Approach to Uropathogenic Escherichia Coli in Urinary Tract Infections" was retracted in 2011. Reason: plagiarized text.

We believe that the methods of detection of the above-mentioned virulence markers are reasonably easy and screening them in a clinical microbiology laboratory is a worthwhile exercise.
